# Clinical Study on Blood Pressure Variability, Montreal Cognitive Assessment and Arteriosclerosis Index in Patients with Cerebral Small Vessel Disease Treated with Integrated Traditional Chinese and Western Medicine by Invigorating Kidney and Removing Blood Stasis

**DOI:** 10.1155/2022/5661303

**Published:** 2022-10-13

**Authors:** Tianzhan Wang, Fang Liang, Yuxin Wang, Qingping Huo, Bing Wang

**Affiliations:** Department of Traditional Chinese Medicine, Shanghai Sixth People's Hospital Affiliated to Shanghai Jiao Tong University School of Medicine, Shanghai 200233, China

## Abstract

**Objective:**

To explore the clinical improvement in blood pressure variability, Montreal Cognitive Assessment, and angiosclerosis index in patients with cerebral small vessel disease treated with integrated traditional Chinese and Western medicine.

**Methods:**

A randomized controlled study of patients with cerebral small vessel disease who were treated in our hospital from November 1, 2018, to January 31, 2022. The enrolled patients were randomized into 2 groups according to the random numbers: an observation group treated with integrated traditional Chinese and Western medicine and a control group treated with Western medicine only. Blood pressure variability, Montreal Cognitive Assessment (MoCA), and angiosclerosis index were compared between the two groups.

**Results:**

There were 71 qualified cases in the observation group and 58 qualified cases in the control group. Before treatment, the indicators between the two groups were comparable (*P* > 0.05). After treatment, the mean values of systolic blood pressure (SBP) and diastolic blood pressure (DBP) were significantly decreased (*P* < 0.05); the decrease of 24hSBP-coefficient of variation (CV), daytime SBP (dSBP)-CV, 24hSBP-standard deviation (SD), and dSBP-SD in the observation group was significantly better than that in the control group; the MoCA scores of the observation group were significantly higher than those of the control group ((*P* < 0.05); the ABI and PWV were significantly different between the two groups (*P* < 0.05); TC, TG, HDL-C, and LDL-C in observation group decreased after treatment, and HDL-C increased significantly (*P* < 0.05).

**Conclusion:**

Integrative traditional Chinese and Western medicine treatment can further reduce the blood pressure variability, especially systolic blood pressure; improve the MoCA score and cognitive function, increase the ankle-brachial index, reduce pulse wave velocity and the degree of arteriosclerosis; and improve lipid metabolism a comprehensive intervention role.

## 1. Introduction

With the aging of the population and changes in people's living habits, the prevalence of stroke in China is increasing year by year, which has become a major social problem. In the past, most of the understanding of cerebral apoplexy was based on two diseases that mainly damage the large blood vessels in the brain, but due to its extensive clinical use, it has been used in many cerebral small vessel diseases (CSVDs) [1–4]. Hypertension and aging are the most important independent risk factors for CSVD, and cognitive impairment and stroke are the final outcomes of the disease. At present, there is a lack of secondary prevention and treatment research on CSVD. Antihypertensive, antithrombotic, and statin lipid regulation are important measures for the treatment of CSVD. Some recent studies have shown that, in addition to blood pressure amplitude, blood pressure variability (BPV) has a significant relationship with the development of CSVD [5]. As a quantitative index, BPV can independently predict changes in the heart, brain, and kidney. Target visceral lesions such as peripheral blood vessels and the risk of cardiovascular disease are the main clinical indicators of CSVD patients. Therefore, early intervention for BPV is very necessary, but there is still a lack of high-level clinical trials to prove it. In this randomized controlled trial (RCT), we analyzed the patients with cerebral small vessel disease treated in our hospital.

## 2. Materials and Methods

This is an RCT of patients with cerebral small vessel disease who were treated at our hospital from November 1, 2018, to January 31, 2022. The subjects were randomized into 2 groups according to the random numbers, one in the observation group (71 cases) and the other in the control group (58 cases); the observation group included 39 males and 32 females, with an average age of (63.24 ± 1.42) years; the control group included 31 males and 27 females, with an average age of (63.89 ± 1.68) years. This study was approved by the Medical Ethics Committee of our hospital (Approval no. 2018–084) and was enrolled in the China Clinical Trial Registry (Registration No. ChiCTR1800018873). The patients and their families were informed and agreed to the study and signed the consent form (Table 1).

### 2.1. Diagnosis, Inclusion, and Exclusion Criteria

- The diagnostic criteria of traditional Chinese medicine (TCM) syndrome types were as follows: (1) dizziness, sore waist, and weak knees; (2) dark purple tongue or ecchymosis; (3) tinnitus, forgetfulness
- Diagnostic criteria were as follows: (1) Clinical manifestations: asymptomatic lacunar infarction, cerebral microbleeds, partial leukoaraiosis, various lacunar syndromes, and vascular cognitive dysfunction; and (2) imaging confirmed as lacunar infarction, perivascular gap enlargement, and white matter lesions
- Inclusion criteria were as follows: (1) met the diagnostic criteria; (2) no macrovascular disease or intracranial tumor; (3) 40–80 years old; (4) MoCA score greater than 26 points; (5) signed informed consent
- Exclusion criteria were as follows: (1) had other cerebral small vessel diseases in the past, such as amyloid angiopathy type, other hereditary disease-related small vessel disease, hypertensive emergency (SBP >180 mmHg, DBP > 110 mmHg), hypertensive crisis, and secondary obesity; (2) severe liver or kidney insufficiency; (3) allergic constitution or allergic to multiple drugs; (4) complicated with other serious diseases

Patients in both groups were treated for 12 weeks. Patients in the control group were given basic medical treatment such as antihypertensive, hypoglycemic, lipid-regulating, and antiplatelet aggregation. Patients in the observation group received the treatments as patients in the control group, combined with the Bushen Huayu Recipe, two doses a day taken in the morning and evening, 200 mL decoction each time. Recipe: 20 g of Cistanche deserticola, 12 g each of Pheretima aspergillum and Alpinia oxyphylla Miq, 10 g each of Salvia miltiorrhiza, and Radix Curcumae.

#### 2.1.1. Observation Indicators Included

- Blood pressure and blood pressure variability including 24 h mean systolic blood pressure (24hSBP), 24 h mean diastolic blood pressure (24hDBP), daytime SBP (dSBP), daytime DBP (dDBP), nighttime SBP (nSBP), nighttime DBP (nDBP), 24 h systolic blood pressure variation (24hSBPv), and 24 h diastolic blood pressure variation (24hDBPv); standard deviation (SD) of 24hSBP (24hSBP-SD), 24hDBP-SD, dSBP-SD, dDBP-SD, nSBP-SD, and nDBP-SD; coefficient of variation (CV; CV = SD/mean) of 24hSBP (24hSBP-CV), 24hDBP-CV, dSBP-CV, dDBP-CV, nSBP-CV, and nDBP-CV, which were detected by ambulatory blood pressure at 0 and 12 weeks of intervention. The respective change levels of subjects before and after intervention and between groups were compared.
- Cognitive function: the Montreal Cognitive Assessment (MoCA Assessment) was assessed at 0 and 12 weeks of the intervention.
- Degree of vascular arteriosclerosis: ankle-brachial index (ABI) and pulse wave velocity (PWV) were examined at 0 and 12 weeks of intervention.
- Serum total cholesterol (TC), triglyceride (TG), high-density lipoprotein cholesterol (HDL-C), and low-density lipoprotein cholesterol (LDL-C) were detected at 0 and 12 weeks of intervention.

### 2.2. Statistical Methods

The data in this experiment were analyzed by SPSS21.0 (SPSS, Chicago, IL, USA), in which the *χ*^*2*^(%) test was performed for the count data, and the *t*-test ($\bar{x}$ ± *s*) was performed for the measurement data. *P* < 0.05 (2-sided) can determine that this experiment has statistical significance.

## 3. Results

There were no significant differences in gender, age, or accompanying diseases between the two groups (*P* > 0.05, Table 1).

### 3.1. Comparison of the Mean Values of 24 h Ambulatory Blood Pressure

Before treatment, there were no significant differences in blood pressure parameters between the two groups (*P* > 0.05). The mean values of systolic blood pressure and diastolic blood pressure in the period after treatment were significantly decreased (*P* < 0.05). There were significantly lower 24hSBP (123.68 ± 3.48 mmHg vs. 130.52 ± 4.38 mmHg) and dSBP (123.62 ± 5.43 mmHg vs. 132.79 ± 6.11 mmHg) in the observation group (*P* < 0.05, Table 2).

### 3.2. Comparison of the Coefficient of Variation (CV) of Ambulatory Blood Pressure

Before treatment, there were no significant differences in the variation coefficients of ambulatory blood pressure between the two groups (*P* > 0.05). After treatment, the 24hSBP-CV, 24hDBP-CV, and dSBP-CV of the two groups decreased significantly (*P* < 0.05). There was a significant decrease in 24hSBP-CV (0.073 ± 0.018 mmHg vs. 0.091 ± 0.020 mmHg) and dSBP-CV (0.059 ± 0.021 mmHg vs. 0.084 ± 0.024 mmHg) in the observation group (*P* < 0.05, Table 3).

### 3.3. Comparison of MoCA Scores between the Two Groups before and after Treatment

There were no differences in MoCA scores between the two groups before treatment (*P* > 0.05). After treatment, the MoCA scores of the observation group were all significantly higher than those of the control group (*P* < 0.05, Table 4).

### 3.4. Comparison of ABI and PWV

Before treatment, there were no significant differences in ABI and PWV between the two groups (*P* > 0.05). After treatment, ABI (1.198 ± 0.081 vs. 1.136 ± 0.077) and PWV (1432.47 ± 191.62 vs. 1523.46 ± 196.73) in the observation group were significantly different than those in the control group (*P* < 0.05, Table 5).

### 3.5. Comparison of TC, TG, HDL-C, and LDL-C

Before treatment, there were no differences in TC, TG, HDL-C, and LDL-C between the two groups (*P* > 0.05). Compared with those before treatment, TC, TG, and LDL-C in the observation group decreased significantly after treatment, and HDL-C increased significantly (*P* < 0.05). Compared with the control group, the LDL-C in the observation group was significantly decreased (*P* < 0.05, Table 6).

## 4. Discussion

CSVD is a clinical cognitive disorder caused by various lesions in the small perforators, arterioles (40–200 um), capillaries, and venules in the brain, with the exception of individual monophyletic disorders. The radiological and pathological features are dispersed. CSVD mainly manifests as cerebral infarction, cerebral hemorrhage, cognitive, emotional, and overall dysfunction, and is mainly characterized by diseases such as lacunar infarction, lacunar infarction, lacunae, white matter, white matter, perivascular space enlargement, and intracerebral microbleeds [6–9]. The vascular lesions of CSVD are microaneurysms, microaneurysms, fatty hyaline degeneration, fibrinoid necrosis, microaneurysms, and hemorrhage of the deep cerebral cortex. The capillaries are tortuous and capillary distribution is significantly reduced.

The epidemiology of CSVD in China is mostly based on cohort studies and community population surveys. Among patients with cerebral infarction in 4 major cities in China, lacunar strokes account for 42.3% of ischemic strokes [10], and 17.2% of the cases were caused by occlusion of small blood vessels [11, 12]. Our department innovatively proposed that the main pathogenesis of CSVD is kidney deficiency and blood stasis based on years of TCM experience and modern medical research. CSVD patients present a gradual decline of vitality after middle age, the disharmony of the five internal organs, the loss of kidney essence and qi, the daily drying up of body water, the emptiness of the sea of marrow, the dystrophy of cerebral collateral circulation, the stasis of brain vessels, the deterioration of visceral functions over time, and the disharmony of qi and blood. Endogenous phlegm and blood stasis intertwine, resulting in atherosclerosis of small cerebral blood vessels, and abnormal vasoconstriction regulation, thus increasing blood pressure and variability. Based on years of experience in the treatment of ischemic cerebrovascular diseases, our TCM recipe is based on kidney deficiency, blood stasis, and phlegm as the target, and we established a TCM recipe consisting of Rou Cong-Rong, leech, Dilong, salvia, turmeric, and Yizhiren, which is a kidney-tonifying and stasis-removing prescription. In the recipe, Rou Cong-Rong tonifies the kidney and strengthens yang, fills the essence, and nourishes the marrow, and the main ingredient is phenylethanoid glycosides, which have antiaging and neuroprotective effects, and improve cognitive function [13, 14]. The leech chases and breaks down bad blood, does not damage fresh blood, and does not damage qi when it enters the blood [15, 16]. Dilong promotes blood circulation and removes blood stasis, dispels wind and clears collaterals, nourishes internal organs, and externally unblocks meridians. The main thrombolytic components can improve microcirculation, which is anticoagulant without affecting hemostasis [17]. Danshen removes bad blood, clears blood vessels, activates blood and removes blood stasis, clears the heart, and removes vexation [18–20]. Curcuma purifies qi, activates blood and dissipates phlegm, nourishes the brain, nourishes the kidney, and tonifies kidney. The combination of various medicines has the effect of invigorating the kidney and removing blood stasis, resolving phlegm, and dredging collaterals. A review of the results of this study showed that the mean value of ambulatory blood pressure and the coefficient of variation of ambulatory blood pressure at each time point in the observation group decreased significantly after treatment, and the MoCA score, ABI, and PWV detection were better than those of the control group. It will be interesting to test the efficacy of Bushen Huayu's integrated traditional Chinese and Western medicine treatment in other diseases affecting the cerebral vessels, such as fulminant hepatitis, hypoxia, and inflammation. [21–30].

In general, Bushen Huayu's integrated traditional Chinese and Western medicine treatment can further reduce the blood pressure variables of CSVD patients, improve the MoCA score and cognitive function, increase the ABI, reduce PWV, reduce the degree of arteriosclerosis, and improve lipid metabolism.

## Figures and Tables

**Table 1:** General information of group 2.

Project	Observation group (*n* = 71)	Control group (*n* = 5)	*t/χ * ^*2*^	*P*
Male/Female (*n*)	39/32	31/27	3.053	0.985
Age (years)	63.24 ± 1.42	63.89 ± 1.68	1.176	0.241
Height (cm)	162.45 ± 11.27	163.83 ± 12.06	4.247	0.805
Weight (kg)	51.62 ± 4.33	52.60 ± 3.95	8.635	0.526
Smoking history	21 (29.58)	15 (25.86)	5.849	0.635
Alcoholism history	17 (23.94)	11 (18.97)	11.273	0.781
Course of disease (years)	3.79 ± 1.03	3.76 ± 1.15	7.492	0.893

Hypertension				
Grade I	25 (35.21)	20 (34.48)	16.845	0.847
Grade II	29 (40.85)	23 (39.66)		
Grade III	17 (23.94)	15 (25.86)		
Diabetes	24 (33.80)	19 (32.76)	9.724	0.846
Coronary heart disease	16 (22.54)	14 (24.14)	2.448	0.751
Hyperlipidemia	64 (90.14)	53 (91.38)	8.729	0.819

**Table 2:** Comparison of 24 h ambulatory blood pressure mean values before and after treatment in the two groups ($\bar{x}$ ± *s*, mmHg).

Group	Observation group (*n* = 71)		Control group (*n* = 58)		*T*	*P* ^#^
	Before therapy	After treatment	Before therapy	After treatment		
24hSBP	146.73 ± 6.23	123.68 ± 3.48^#^	145.96 ± 6.34	130.52 ± 4.38^#^	7.482	0.035
24hDBP	81.56 ± 7.16	72.27 ± 6.33^#^	79.82 ± 8.36	71.36 ± 6.27^#^	4.394	0.873
dSBP	148.71 ± 8.43	123.62 ± 5.43^#^	147.82 ± 8.49	132.79 ± 6.11^#^	11.751	0.005
dDBP	81.57 ± 7.39	73.89 ± 6.28^#^	82.25 ± 7.42	72.43 ± 6.45^#^	8.463	0.497
nSBP	137.64 ± 17.58	122.89 ± 9.71^#^	138.39 ± 13.25	125.89 ± 9.06^#^	10.527	0.693
nDBP	77.34 ± 10.83	69.47 ± 7.56^#^	76.92 ± 9.68	67.89 ± 7.49^#^	15.263	0.749

*Note.* ^#^Comparison between groups after treatment.

**Table 3:** Comparison of the coefficient of variation of ambulatory blood pressure before and after treatment in the two groups ($\bar{x}$ *±* *s*, mmHg).

Group	Observation group (*n* = 71)		Control group (*n* = 58)		*T*	*P* ^#^
	Before therapy	After treatment	Before therapy	After treatment		
24hSBP-CV	0.117 ± 0.053	0.073 ± 0.018^#^	0.115 ± 0.046	0.091 ± 0.020^#^	8.347	0.035
24hDBP-CV	0.132 ± 0.195	0.119 ± 0.025^#^	0.126 ± 0.103	0.098 ± 0.021^#^	6.559	0.376
dSBP-CV	0.113 ± 0.035	0.059 ± 0.021^#^	0.115 ± 0.041	0.084 ± 0.024^#^	11.548	0.015
dDBP-CV	0.124 ± 0.043	0.105 ± 0.029	0.122 ± 0.038	0.113 ± 0.033	9.325	0.579
nSBP-CV	0.122 ± 0.194	0.085 ± 0.031	0.123 ± 0.096	0.087 ± 0.028	13.739	0.417
nDBP-CV	0.119 ± 0.042	0.115 ± 0.036	0.121 ± 0.043	0.117 ± 0.041	7.681	0.689

*Note.* ^#^Comparison between groups.

**Table 4:** Comparison of MoCA scores between the two groups before and after treatment ($\bar{x}$*± s*, score).

Group	Observation group (*n* = 71)		Control group (*n* = 58)		*t*	*P* ^#^
	Before therapy	After treatment	Before therapy	After treatment		
Total score	16.83 ± 4.07	22.35 ± 6.23^#^	16.49 ± 4.13	18.15 ± 4.64	9.547	<0.001
Verbal fluency	0.95 ± 0.24	5.69 ± 1.34^#^	0.89 ± 0.23	3.12 ± 0.87^#^	11.619	0.005
Naming	1.21 ± 0.31	5.26 ± 1.31^#^	1.23 ± 0.36	3.39 ± 0.92^#^	8.539	0.003
Abstraction	0.83 ± 0.25	1.96 ± 0.42^#^	0.82 ± 0.24	1.09 ± 0.38	6.247	0.031
Attention	2.97 ± 0.63	5.89 ± 1.27^#^	3.04 ± 0.61	4.12 ± 1.03	16.394	0.015
Delayed recall	0.97 ± 0.33	4.15 ± 0.82^#^	0.93 ± 0.31	1.25 ± 0.49	7.132	0.001
Orientation score	2.46 ± 0.42	5.26 ± 0.91^#^	2.44 ± 0.39	3.51 ± 0.46	8.429	0.035
Visuoconstructional skills	1.77 ± 0.46	5.38 ± 1.29^#^	1.81 ± 0.46	2.41 ± 0.59	13.762	<0.001

*Note.* ^#^Comparison between groups.

**Table 5:** Comparison of ABI and PWV between the two groups before and after treatment ($\bar{x}$*± s*).

Group	Observation group (*n* = 71)		Control group (*n* = 58)		*T*	*P*
	Before therapy	After treatment	Before therapy	After treatment		
ABI	1.093 ± 0.074	1.198 ± 0.081^#^	1.094 ± 0.071	1.136 ± 0.077^#^	9.547	0.045
PWV	1661.53 ± 206.24	1432.47 ± 191.62^#^	1660.47 ± 204.23	1523.46 ± 196.73^#^	11.619	<0.001

*Note.* ^#^Comparison between groups.

**Table 6:** Comparison of TC, TG, HDL-C, and LDL-C between the two groups before and after treatment ($\bar{x}$ ± *s*, _mmol/L_).

Group	Observation group (*n* = 71)		Control group (*n* = 58)		*T*	*P* ^#^
	Before therapy	After treatment	Before therapy	After treatment		
TC	4.88 ± 1.18	4.01 ± 0.92^#^	4.85 ± 1.14	3.95 ± 0.87^#^	10.271	0.642
TG	1.64 ± 0.59	1.08 ± 0.41^#^	1.62 ± 0.56	1.12 ± 0.38^#^	8.446	0.703
HDL-C	1.18 ± 0.45	1.43 ± 0.67^#^	1.19 ± 0.46	1.28 ± 0.52^#^	6.382	0.492
LDL-C	2.91 ± 0.93	1.91 ± 0.36^#^	2.93 ± 0.97	2.25 ± 0.74^#^	9.734	0.035

*Note.* ^#^Comparison between groups.

## Data Availability

The data used to support the findings of this study are available from the corresponding author upon request.
